# HOXC6: A promising biomarker linked to an immunoevasive microenvironment in colorectal cancer based on TCGA analysis and cohort validation

**DOI:** 10.1016/j.heliyon.2023.e23500

**Published:** 2023-12-10

**Authors:** Meilin Weng, Yuling Lai, Xiaodong Ge, Wenchao Gu, Xixue Zhang, Lihong Li, Minli Sun

**Affiliations:** a Department of Anesthesiology, Zhongshan hospital, Fudan University, Shanghai, 200032, China; b Shanghai Key Laboratory of Perioperative Stress and Protection, Zhongshan hospital, Fudan University, Shanghai, 200032, China; c Department of Diagnostic and Interventional Radiology, University of Tsukuba, Faculty of medicine, Ibaraki, Tsukuba, Japan; d Department of Anesthesiology, Huadong Hospital Affiliated to Fudan University, No 221, West Yan'an Road, Shanghai 200040, China; e Department of Anesthesiology, Shanghai Cancer Center, Fudan University, Shanghai, 200032, China

**Keywords:** *HOXC6*, Biomarker, Immunoevasive, tumor microenvironment, Colorectal cancer, TCGA

## Abstract

*HOXC6* plays an essential part of the carcinogenesis of solid tumors, but its functional relevance within the immune contexture in patients with colorectal cancer (CRC) is still uncertain. We intended to investigate the predictive value of *HOXC6* expression for survival outcomes and its correlation with immune contexture in CRC patients by utilizing the Cancer Genome Atlas database (n = 619). Validation was performed in cohorts from Zhongshan Hospital (n = 200) and Shanghai Cancer Center (n = 300). Immunohistochemical (IHC) staining was utilized to compare the levels of immunocytes infiltrating the tumor between the groups with high and low expression of *HOXC6*. Elevated levels of *HOXC6* expression in CRC tissues were linked to malignant progression and poor prognosis. *HOXC6* as a risk factor for survival of CRC patients was confirmed. Receiver operating characteristic analysis confirmed its diagnostic value, and a reliable prognostic nomogram was constructed. KEGG analysis and GSEA showed that *HOXC6* participated in immune regulation, and its expression was tightly linked to the abundance of infiltrating immunocytes. *HOXC6* was upregulated in patients diagnosed with CRC within the two cohorts, and high *HOXC6* levels were correlated with a worse prognosis. The high-*HOXC6* expression group showed increased infiltration of Treg cells, CD68^+^ macrophages, CD66b^+^ neutrophils, and CD8^+^ T-cells and elevated levels of PD-L1 and PD-1, but decreased levels of granzyme B and perforin. These findings suggest that *HOXC6* abundance in patients with CRC determines a poor prognosis, promotes an immunoevasive environment, and directs CD8^+^ T-cell dysfunction. *HOXC6* is expected to become a prospective biomarker for the outcome of CRC.

## Abbreviations

HOXC6: Homeobox C6
CRC: colorectal cancer
TCGA: The Cancer Genome Atlas
GEO: Gene Expression Omnibus
KEGG: Kyoto Encyclopedia of Genes and Genomes
GSEA: gene set enrichment analysis
AUC: area under curve
ROC: receiver-operating characteristic
PPI: Protein-protein interaction
GO: Gene Ontology
IHC: Immunohistochemical
GZMB: granzyme B
PRF1: perforin
PD-L1: programmed cell death-ligand 1
PD-1: programmed cell death protein 1
TME: tumor microenvironment
OS: overall survival
PFI: progression-free interval
DSS: disease-specific survival
RT-qPCR: quantitative reverse transcription PCR
ICB: immune checkpoint blockade
CTLA-4: Cytotoxic T-Lymphocyte Associated Antigen 4
dMMR: defective DNA mismatch repair

## 1 Introduction

Colorectal cancer (CRC) is the second highest contributor to cancer-related fatalities in the United States, with over 1.9 million new cases reported worldwide in 2020 [1,2]. Although its overall incidence has begun to stabilize or decrease annually in some developed countries, its morbidity and mortality have begun to show an increasing annual trend in individuals aged <50 years. In this age group, the disease tends to reach a severe clinical stage, affect distant organs, and exhibit a high recurrence rate [3]. China, the world's largest developing country, bears a substantial burden of cancer. China is currently undergoing a transition in its cancer landscape, with changes mirroring the shift observed in cancer patterns from developing to developed nations. The incidence and mortality rates of CRC, prostate cancer and breast cancer are rising rapidly [4,5]. Current treatments for CRC include surgery (primary and metastatic lesions), radiotherapy, and chemotherapy [6]. Nevertheless, there has been minimal advancement in the 5-year survival rate for patients diagnosed with CRC over the recent years. Consequently, there is an imperative need to find novel biomarkers for early disease detection and promising therapeutic targets to extend patient survival.

The *HOX* gene family determines vertebrate morphogenesis and embryonic development by encoding highly conserved transcription factors. Recent evidence has shown that certain members within the *HOX* group are instrumental in the advancement of various solid tumors [7], including bladder, lung [8], prostate [9], and breast tumors [10]. The *HOX* group, comprising *HOXA*, *HOXB*, *HOXC*, and *HOXD* [11], is responsible for cancer-related biological behaviors [12]. *HOXA*, *HOXB*, *HOXC*, and *HOXD* are primarily highly expressed in patients with ovarian, colon, prostate, and breast cancer, respectively [13]. However, only a few studies have examined *HOXC* in CRC. The *HOXC* gene family includes *HOXC4*, *HOXC5*, *HOXC6*, *HOXC8*, *HOXC9*, *HOXC10*, *HOXC11*, *HOXC12*, and *HOXC13*, which are situated on chromosome 12q13.3. Among these, *HOXC11*, which is enormously expressed in CRC, is closely linked to the overall survival (OS) of patients [14]. Studies on its underlying mechanism suggest that *HOXC11* might promote the progression of CRC cells through the peroxisome proliferator-activated receptor. In addition, the overexpression of *HOXC13* in esophageal squamous cell carcinoma is closely related to worse outcome, with *HOXC13* knockdown inhibiting the proliferation of esophageal squamous epithelial cells in vitro [15]. Nevertheless, the expression and prognostic importance of *HOXC6* in patients diagnosed with CRC are still not clear. One study found that the downregulation of *HOXC6* in HCT116 CRC cells can suppress tumor cell proliferation by inhibiting the autophagy pathway [16]. This work suggested *HOXC6* as a potential therapeutic marker, but without further clinical verification. Qi et al. [17] suggested that elevated *HOXC6* level was strongly correlated to the cytokine pathway, immune cell infiltration rate, T-cell chemokine expression and immune checkpoint expression. However, this study lacked comprehensive evaluation and clinical cohort validation. Further exploration of the roles and functional relevance of *HOXC6* in the immune context of patients with CRC is required to gain crucial insights.

This study utilized the information from The Cancer Genome Atlas (TCGA) database to detect *HOXC6* levels in patients diagnosed with CRC and investigate its expression in relation to clinical prognosis (clinicopathological parameters and outcome). In addition, Kyoto Encyclopedia of Genes and Genomes (KEGG) analysis and gene set enrichment analysis (GSEA) were employed to identify biological pathways associated with *HOXC6* in CRC. Immune infiltration analysis by single-sample GSEA (ssGSEA) was adopted to estimate the relevance between *HOXC6* levels and immune infiltration in patients diagnosed with CRC. We additionally verified the level, clinical significance, and immune relevance of *HOXC6* in two cohorts from Zhongshan Hospital and Shanghai Cancer Center. The results of this study emphasize that *HOXC6* may be a prospective biomarker and curative target for CRC. Furthermore, these detections can offer a novel view on the impact of *HOXC6* on the tumor immune microenvironment and reveal its potential function in CRC progression.

## 2 Results

### 2.1 *HOXC6* was upregulated in CRC tissues

As shown in Supplementary Table 1, we downloaded the clinical characteristics and gene expression records of 619 colorectal cancers from TCGA and used them in this study. The median diagnosis age was 68. Patient distribution included 105 in stage I, 227 in stage II, 179 in stage III, and 88 in stage IV. Most tumors (73.3 %, n = 454) were colon adenocarcinomas, while 26.7 % (n = 165) were rectal adenocarcinomas.

Utilizing the Wilcoxon signed-rank test (Fig. 1), we conducted a comparison of *HOXC6* expression in 619 CRC tissues and 51 normal tissues. The level of *HOXC6* in the tumor tissues was dramatically raised compared to the normal tissues (P = 0.036; Fig. 1A). The Wilcoxon signed-rank test was employed to study the level of *HOXC6* in 50 paired CRC tissues and their paired normal tissues. The findings indicated that the relative expression of *HOXC6* in 50 CRC tissues was markedly higher than that in the 50 matched normal tissues (P < 0.001, Fig. 1B). Using the Wilcoxon rank-sum test, we contrasted the level of *HOXC6* in normal tissues of Genotype-Tissue Expression (GTEx) combined with TCGA and tumor tissues solely from TCGA (Fig. 1C, p = 0.503). Moreover, *HOXC6* exhibited significant expression in numerous malignancies (Fig. 1D), such as bladder urothelial carcinoma, esophageal cancer, cervical squamous cell carcinoma, glioblastoma multiforme, lung squamous cell carcinoma, stomach adenocarcinoma, sarcoma, prostate adenocarcinoma, etc.

**Fig. 1:** ***HOXC6* is elevated in CRC tissues and is related to malignant progression**. (**A)***HOXC6* expression levels in 51 healthy and 619 tumor tissues. **(B)***HOXC6* expression levels in 50 CRC and their paired normal tissues. **(C)***HOXC6* expression in normal samples of GTEx combined with those obtained from TCGA and tumor samples from TCGA (P = 0.503). **(D)** Human *HOXC6* expression levels in different cancers obtained from the TCGA database. **(E**–**J)** Association between elevated *HOXC6* expression and clinical pathological characteristics, including T stage, N stage, neoplasm type, pathological stage, TP53 status, and BRAF status (all P < 0.05). *P < 0.05, **P < 0.01, or ***P < 0.001 were considered significant differences.

### 2.2 Relationship between upregulation of *HOXC6* gene expression and the advancement and outcome of patients with CRC

*HOXC6* was expressed in 619 CRC samples, and the associated data were studied using the TCGA database. After the Wilcoxon signed-rank test and Kruskal-Wallis test, increased expression of *HOXC6* in CRC samples was markedly linked to T stage (P < 0.001), N stage (P = 0.022), neoplasm type (P < 0.001), pathological state (P = 0.028), TP53 status (P < 0.001), and BRAF status (P < 0.001; Fig. 1E–J). There was no notable association found between these elevated levels of *HOXC6* and the M stage, CEA level, history of colon polyps, presence of colon polyps, or KRAS status (all P > 0.05, Supplementary figs. 1A–E).

To explore the function of *HOXC6* in CRC additionally, we analyzed the relevance between the expression of *HOXC6* and the clinicopathological features of patients diagnosed with CRC using the TCGA dataset. The cutoff value was determined according to the median expression level. Notably, elevated expression of *HOXC6* was closely linked to T stage (P < 0.001), lymph node metastasis (P = 0.014), neoplasm type (P < 0.001), TP53 status (P = 0.002), BRAF status (P < 0.001), and age (P = 0.038) but not with sex, CEA level, history of colon polyps, KRAS status, presence of colon polyps, distant metastasis, or pathological stage (all P > 0.05) (Table 1).

**Table 1:** Relevance between *HOXC6* level and the clinicopathological features of patients diagnosed with CRC from TCGA.

Characters	level	Low expression of *HOXC6*	High expression of *HOXC6*	P value
n		310	309	
T stage (%)	T1	14 (4.5 %)	6 (1.9 %)	0.001
	T2	63 (20.4 %)	42 (13.6 %)	
	T3	210 (68.0 %)	212 (68.8 %)	
	T4	22 (7.1 %)	48 (15.6 %)	
N stage (%)	N0	182 (58.9 %)	169 (55.0 %)	0.014
	N1	83 (26.9 %)	67 (21.8 %)	
	N2	44 (14.2 %)	71 (23.1 %)	
M stage (%)	M0	233 (86.0 %)	226 (82.2 %)	0.274
	M1	38 (14.0 %)	49 (17.8 %)	
Pathological stage (%)	Stage I	62 (20.8 %)	43 (14.3 %)	0.165
	Stage II	108 (36.2 %)	119 (39.5 %)	
	Stage III	89 (29.9 %)	90 (29.9 %)	
	Stage IV	39 (13.1 %)	49 (16.3 %)	
Sex (%)	Female	147 (47.4 %)	142 (46.0 %)	0.776
	Male	163 (52.6 %)	167 (54.0 %)	
CEA level (%)	≤5	128 (62.7 %)	124 (64.2 %)	0.836
	>5	76 (37.3 %)	69 (35.8 %)	
History of colon polyps (%)	NO	193 (70.4 %)	171 (66.3 %)	0.348
	YES	81 (29.6 %)	87 (33.7 %)	
Colon polyps present (%)	NO	97 (70.8 %)	110 (68.3 %)	0.736
	YES	40 (29.2 %)	51 (31.7 %)	
Neoplasm type (%)	Colon adenocarcinoma	190 (61.3 %)	264 (85.4 %)	<0.001
	Rectum adenocarcinoma	120 (38.7 %)	45 (14.6 %)	
TP53 status (%)	Mut	170 (66.1 %)	142 (52.8 %)	0.002
	WT	87 (33.9 %)	127 (47.2 %)	
KRAS status (%)	Mut	96 (37.4 %)	118 (43.9 %)	0.152
	WT	161 (62.6 %)	151 (56.1 %)	
BRAF status (%)	Mut	6 (2.3 %)	61 (22.7 %)	<0.001
	WT	251 (97.7 %)	208 (77.3 %)	
Age (%)	≤65	148 (47.7 %)	121 (39.2 %)	0.038
	>65	162 (52.3 %)	188 (60.8 %)	

We then assessed the relevance between *HOXC6* expression and the outcome of patients diagnosed with CRC. Increased *HOXC6* expression was linked to worse OS (hazard ratio [HR]: 1.68; 95 % confidence interval [CI]: 1.18–2.40; P = 0.004), disease-specific survival (DSS) (HR: 1.97; 95 % CI: 1.24–3.14; P = 0.004), and progression-free interval (PFI) (HR: 1.53; 95 % CI: 1.11–2.09; P = 0.008) (Fig. 2A–C). Overall, these findings suggested that increased *HOXC6* level was linked to the outcome of patients diagnosed with CRC.

**Fig. 2:** The upregulation of *HOXC6* is related to poorer survival, and *HOXC6* is a promising risk factor for CRC. **(A**–**C)** Increased *HOXC6* expression was related to poorer overall survival (OS), disease-specific survival (DSS), and progression-free interval (PFI). (**D–F)** Uni- and multivariate Cox analyses of *HOXC6* expression and other clinical pathological variables in OS, DSS, and PFI.

The relevance between *HOXC6* expression and clinicopathological features was studied using logistic regression analysis. Increased *HOXC6* expression in patients with CRC was prominently associated with advanced T stage (odds ratio [OR] = 1.80 [1.21–2.70], P = 0.004), colon adenocarcinoma (OR = 0.27 [0.18–0.40], P < 0.001), wild-type TP53 status (OR = 0.57 [0.40–0.81], P = 0.002), and mutant BRAF status (OR = 12.27 [5.62–32.27], P < 0.001) (Supplementary Table 2).

We analyzed the predictive factors for OS using both univariate and multivariate Cox regression methods (Fig. 2D, Supplementary Table 3). High *HOXC6* expression (HR: 3.268; 95 % CI, 1.775–6.018; P < 0.001), age (HR: 3.624; 95 % CI, 1.903–6.900; P < 0.001), distant metastasis (HR: 3.057; 95 % CI, 1.413–6.614; P = 0.005), and pathological stage (HR: 5.049; 95 % CI, 1.163–21.917; P = 0.031) were risk factors correlated with poor OS, suggesting that high *HOXC6* levels are related to worse outcome. We also analyzed the predictive factors for PFI and DSS (Fig. 2E and F, Supplementary tables 4–5), and the outcome indicated that *HOXC6* expression was independently related to DSS (HR: 3.357; 95 % CI: 1.693–6.655; P < 0.001) and PFI (HR: 2.810; 95 % CI: 1.636–4.828; P < 0.001).

To further estimate the effectiveness of *HOXC6* as a biomarker for CRC, we examined the AUC values in the ROC curve for OS, DSS, and PFI at 1, 3, and 5 years (Fig. 3A–C). *HOXC6* possessed a strong prognostic capability in patients with CRC (3-year: OS-AUC: 0.666; DSS-AUC: 0.699; PFI-AUC: 0.632).

**Fig. 3:** The prognostic value of *HOXC6* and the nomogram based on *HOXC6* expression in predicting the prognosis of patients with CRC. (**A–C)** ROC was employed to predict the impact of *HOXC6* expression on OS, DSS, and PFl in patients with CRC at 1, 3, and 5 years. **(D**–**F)** A nomogram according to *HOXC6* expression, age, CEA level, pathological stage, KRAS status, and M stage was built to forecast the OS, DSS, and PFI in patients with CRC at 1, 3, and 5 years. **(G**–**I)** 1-, 3-, and 5-year calibration curves for OS, DSS, and PFI in patients with CRC.

### 2.3 Construction of a nomogram based on *HOXC6* expression

To forecast the likelihood of survival for patients with CRC over 1, 3, and 5 years, a nomogram was constructed to visually depict the relationships among six clinicopathological variables (*HOXC6* expression, age, CEA level, pathological stage, M stage, and KRAS status). The nomogram's C-index values were 0.806, 0.831, and 0.747 for OS, DSS, and PFI, respectively, indicating a moderate level of predictive accuracy (Fig. 3D–F). The calibration curves for 1, 3, and 5 years indicated that our outcomes were consistent with the predicted values. The nomogram based on *HOXC6* expression was thus considered to be satisfactory (Fig. 3G–I).

### 2.4 Networks of interactions between proteins (PPI) and enrichment analysis

We employed STRING for PPI network analysis to explore the coregulatory proteins associated with *HOXC6*, in which the *HOXC6*-related genes included *HOXA6*, *HOXB5*, *HOXB4*, *HOXB6*, *HOXA5*, *HOXA7*, *HOXC5*, *HOXC4*, and *HOXD4*. All scores were above 0.9 (Fig. 4A). To forecast the performance of *HOXC6*, along with its related pathways, we identified the first 300 positively coexpressed *HOXC6* genes from the TCGA database. Fig. 4B shows the first 20 genes. Through enrichment analysis on the top 300 genes that are highly associated with *HOXC6*, the probable biological functions and functional pathways of *HOXC6* were further investigated. Gene Ontology (GO) and KEGG pathway analyses showed that high *HOXC6* expression was concentrated in the cell adhesion molecule pathway (Fig. 4C and D). We also employed GSEA to investigate the biological pathways associated with high *HOXC6* expression. Our results revealed that a phenotype characterized by high *HOXC6* expression comprised many key pathways and was correlated with tumorigenesis. In the high-*HOXC6* expression group, noteworthy pathways enriched involved neutrophil degranulation, receptor tyrosine kinase signaling, GPCR ligand binding, neuronal systems, G alpha I signaling events, and pathways in cancer (Supplementary Table 6). Fig. 4E shows the most significantly enriched neutrophil degranulation pathway on the basis of the normalized enrichment score (NES). Fig. 4F and Supplementary Table 7 show other significant GSEA results pertaining to the expression of the top 300 genes most closely linked to *HOXC6*. The results revealed that immunoregulatory interactions between lymphoid and nonlymphoid cells, KEGG cytokine receptor interactions, and reactome extracellular matrix organization were also considerably enriched. Thus, KEGG analysis and GSEA showed that *HOXC6* was involved in immune regulation.

**Fig. 4:** PPI networks and enrichment analysis of *HOXC*6. (A) STRING was used to analyze *HOXC6* and its potential coregulatory gene networks. **(B)** The top 20 most positively coexpressed genes of *HOXC6* from analyzing TCGA data are shown in a heatmap. **(C**–**D)** GO (including BP, CC, and MF) and KEGG enrichment for *HOXC6* in CRC samples. **(E)** The results of representative GSEA show that *HOXC6* was concentrated in the neutrophil degranulation pathway. **(F)** Other important GSEA results of the first 300 genes most positively correlated with *HOXC6* expression using a ridge plot, including KEGG and Reactome pathways.

### 2.5 Relationship between *HOXC6* expression and immune infiltration

Fig. 5A shows a significant relevance between *HOXC6* level and increased presence of immunocytes, including macrophages, Th1 cells, cytotoxic cells, NK cells, activated dendritic cells and immature dendritic cells. Subsequently, the Spearman correlation and Wilcoxon signed-rank test were utilized to examine the relationship between *HOXC6* level and the abundance of infiltrating macrophages, neutrophils, CD8^+^ T-cells, mast cells, cytotoxic cells, Tregs, and immune checkpoint genes (Fig. 5B, D–K). The findings indicated that increased *HOXC6* expression was strongly linked to high levels of infiltrating immunocytes and immune checkpoint genes (PD-1, LAG3, and CTLA-4). We also assessed the correlation between the abundance of 10 immunocytes in patients diagnosed with CRC. Fig. 5C's heatmap exhibits a strong correlation among the proportions of different tumor-infiltrating immune cells.

**Fig. 5:** Relationship between *HOXC6* expression and immune infiltration. (A**)***HOXC6* expression is markedly related to dominant immunocyte infiltration in the TCGA cohort. **(B)** The Wilcoxon signed-rank test was employed to identify the level of immunocyte infiltration in the *HOXC6* high/low-expression groups. **(C)** Correlation between the abundance of ten infiltrating immunocytes in patients with CRC. **(D**–**K)** Spearman correlation was employed to calculate the association between *HOXC6* expression and the levels of infiltrating immunocytes (Treg, CD8^+^ T-cells, neutrophils, macrophages, and mast cells) and immune checkpoint molecules (PD-1, CTLA-4, and LAG3). *P < 0.05, **P < 0.01, and ***P < 0.001 were considered significant differences compared to the low-*HOXC6* expression group.

### 2.6 *HOXC6* expression was increased in CRC tissues during clinical validation

We explored the level of *HOXC6* in both CRC tissues and noncancerous tissues of the Zhongshan Hospital cohort using western blotting and quantitative reverse transcription PCR **(**RT‒qPCR) techniques. The protein expression of *HOXC6* was markedly elevated in CRC tissues compared to noncancerous tissues (Fig. 6A and B). The relative expression of *HOXC6* mRNA in both cancerous and noncancerous tissues (n = 80) were identical to the observed protein expression of *HOXC6* (Fig. 6C). The validity of these findings was verified again in the Shanghai Cancer Center cohort (Supplementary figs. 2A–C).

**Fig. 6:** *HOXC6* abundance determines poor prognosis, facilitates an immunoevasive environment, and damages CD8^+^ T-cell function in CRC. (A**)** In the Zhongshan Hospital cohort, *HOXC6* protein expression in CRC and noncancerous tissues was detected using western blotting. T: cancer tissue; N: noncancerous tissues. **(B)** In the Zhongshan Hospital cohort, the relative expression of *HOXC6* in cancer tissue was normalized to β-actin expression and is shown as the fold-change compared with noncancerous tissue (cancer tissue vs. noncancerous tissue, P = 0.0004). **(C)** In the Zhongshan Hospital cohort, RT‒qPCR was employed to detect the relative expression of *HOXC6* mRNA in CRC and noncancerous tissues (n = 80, P < 0.0001). **(D)** OS curves between the high- and low-*HOXC6* expression groups in the Zhongshan Hospital cohort. Blue: low *HOXC6* group; green: high *HOXC6* group. **(E**–**H)** Representative IHC staining images of four major tumor-infiltrating immunocyte subtypes in the high- and low-*HOXC6* expression groups, namely, Foxp3^+^ Treg cells, CD8^+^ T-cells, CD68^+^ macrophages, and CD66b^+^ neutrophils. Scale bar: 250 μm. **(I**–**L)** IHC staining showed typical images of effector molecules (GZMB, PRF1) and immune checkpoint molecules (PD-L1, PD-1) between the two groups. Scale bar: 250 μm. **(M**–**T)** The levels of Foxp3^+^ Treg cells, CD8^+^ T-cells, CD68^+^ macrophages, CD66b^+^ neutrophils, effector molecules (GZMB, PRF1), and immune checkpoint molecules (PD-L1, PD-1) were compared between the two groups. *P < 0.05, **P < 0.01, and ***P < 0.001 were considered significant differences compared to the low-*HOXC6* expression group. (For interpretation of the references to color in this figure legend, the reader is referred to the Web version of this article.)

### 2.7 The group with elevated *HOXC6* expression under clinical validation, which revealed a correlation with malignant progression, an unfavorable prognosis, and an immunoevasive environment

To assure the clinical importance of *HOXC6* in CRC, we assessed the relevance between the levels of *HOXC6* (high/low) and the clinicopathological features of CRC patients from Zhongshan Hospital (n = 200, low *HOXC6* n = 126; high *HOXC6* n = 74). We took the median mRNA expression of *HOXC6* as the cutoff value. The high-*HOXC6* expression group showed a strong association with right-sided colon cancer, poor differentiation, positive surgical margins, nerve invasion, the presence of one or more cancer nodules, and a severe pathological stage (Table 2). In the Shanghai Cancer Center cohort (n = 300; low *HOXC6* expression: n = 216; high *HOXC6* expression: n = 84), high *HOXC6* expression was significantly associated with an age of ≤54, right-sided colon cancer, poor differentiation, positive surgical margins, nerve invasion, the presence of one or more cancer nodules, and severe pathological stage (Supplementary Table 8). Our study indicated that elevated *HOXC6* expression was closely related to the progression of malignant tumors.

**Table 2:** Relevance between *HOXC6* level and the clinicopathological features of the Zhongshan Hospital cohort patients.

Characters	level	Low *HOXC6* group	High *HOXC6* group	P value
n		126	74	
Age, n (%)	≤44	11 (8.7 %)	12 (16.2 %)	0.434
	45–54	19 (15.1 %)	13 (17.6 %)	
	55–64	43 (34.1 %)	23 (31.1 %)	
	65–74	36 (28.6 %)	20 (27.0 %)	
	≥75	17 (13.5 %)	6 (8.1 %)	
Gender, n (%)	Female	81 (64.3 %)	51 (68.9 %)	0.504
	Male	45 (35.7 %)	23 (31.1 %)	
Tumor location, n (%)	Rectum	65 (51.6 %)	38 (51.4 %)	0.018
	Left-side colon	35 (27.8 %)	10 (13.5 %)	
	Right-side colon	26 (20.6 %)	26 (35.1 %)	
Tumor differentiation, n (%)	Well	4 (3.2 %)	0 (0 %)	<0.001
	Moderate	87 (69.0 %)	34 (45.9 %)	
	Poor Unknown	24 (19.0 %) 11 (8.7)	39 (52.7 %) 1 (1.4)	
Tumor histology, n (%)	adenocarcinoma	109 (86.5 %)	61 (82.4 %)	0.071
	ucoid adenocarcinoma	15 (11.9 %)	7 (9.5 %)	
	signet-ring cell carcinoma	2 (1.6 %)	6 (8.1 %)	
Positive Surgical margin, n (%)	No	125 (99.2 %)	67 (90.5 %)	0.003
	Yes	1 (0.8 %)	7 (9.5 %)	
Nerve invasion	No	103 (81.7 %)	42 (56.8 %)	<0.001
	Yes	23 (18.3 %)	32 (43.2 %)	
Infiltrating lymph nodes>12, n (%)	No	28 (22.2 %)	23 (31.1 %)	0.165
	Yes	98 (77.8 %)	51 (68.9 %)	
Number of cancer nodule≥1，n (%)	No	106 (84.1 %)	42 (56.8 %)	<0.001
	Yes	20 (15.9 %)	32 (43.2 %)	
Pathological stage, n (%)	Stage I	18 (14.3 %)	1 (1.4 %)	<0.001
	Stage II	41 (32.5 %)	4 (5.4 %)	
	Stage III	46 (36.5 %)	47 (63.5 %)	
	Stage IV Unkown	15 (11.9 %) 6 (4.8 %)	22 (29.7 %) 0 (0.0 %)	

To further study the correlation between high/low *HOXC6* levels and the clinical outcomes of 200 patients with CRC from Zhongshan Hospital, we utilized Kaplan-Meier analysis. We found that patients diagnosed with CRC and exhibiting elevated levels of *HOXC6* expression had poor OS compared to those with lower *HOXC6* expression (P = 0.005; log-rank test; Fig. 6D). Similarly, within the Shanghai Cancer Center cohort (n = 300), the high-*HOXC6* expression group exhibited inferior OS (P = 0.016; determined by log-rank test; Supplementary Fig. 2D). In summary, high *HOXC6* expression was closely linked to inferior OS in patients diagnosed with CRC.

We conducted immunohistochemical (IHC) staining on tumor-infiltrating immunocytes within the high- and low-*HOXC6* expression groups (n = 20) to explore the underlying mechanism of *HOXC6* in CRC progression. The high-*HOXC6* expression group exhibited elevated levels of Foxp3^+^ Treg cells, CD68^+^ macrophages, CD66b^+^ neutrophils, and CD8^+^ T-cells (Fig. 6E–H, 6M−P, all P < 0.01), indicating an immunosuppressive TME. We further investigated whether increased *HOXC6* expression could affect the role of CD8^+^ T-cells. The elevated-*HOXC6* expression group exhibited reduced expression of GZMB and PRF1 but increased level of PD-L1 and PD-1 compared with the low-*HOXC6* expression group (Fig. 6I–L, 6Q–T, all P < 0.01). In summary, high *HOXC6* expression could potentially indicate a microenvironment for immune evasion and promote CD8^+^ T-cell dysfunction in patients diagnosed with CRC.

To verify the findings shown in Fig. 3D, we constructed a nomogram with five clinicopathological variables (*HOXC6* expression, age, CEA level, pathological stage, and M stage) from the Zhongshan Hospital cohort to forecast the likelihood of survival for patients diagnosed with CRC over 1, 3, and 5 years. The OS C-index was 0.628, indicating moderate prediction accuracy (Supplementary Fig. 3A). The nomogram displayed a robust prognostic capability for patients diagnosed with CRC, with an AUC of 0.661 for 1-year OS, 0.677 for 3-year OS, and 0.643 for 5-year OS (Supplementary Fig. 3B). Furthermore, the calibration curves for 1, 3, and 5 years indicated that our outcomes were consistent with the predicted values (Supplementary Fig. 3C). Therefore, the nomogram based on *HOXC6* expression within the Zhongshan Hospital cohort was considered to be satisfactory.

## 3 Discussion

Using bioinformatics analysis based on TCGA data, our analysis uncovered that *HOXC6* is excessively expressed in CRC and is linked to malignant advancement and an unfavorable prognosis. The results validated *HOXC6* as a hazard factor for OS, PS, and DSS among patients diagnosed with CRC, and ROC analysis confirmed its diagnostic value. We successfully constructed a nomogram based on *HOXC6* expression and other variables, demonstrating satisfactory performance. In addition, GSEA revealed that pathways such as neutrophil degranulation, immunoregulatory interactions between lymphoid and nonlymphoid cells, and cytokine receptor interaction signaling were enriched in the high-*HOXC6* expression phenotype. Further findings indicated that *HOXC6* expression was strongly linked to the infiltration of various immunocyte categories, including Tregs, neutrophils, macrophages, mast cells, and CD8^+^ T-cells. According to TCGA data analysis, it can be inferred that *HOXC6* serves as latent marker and a promising treatment target for CRC.

In the Zhongshan Hospital and Shanghai Cancer Center cohorts, we used western blotting and RT‒qPCR to confirm the upregulation of *HOXC6* in patients diagnosed with CRC. Our results found that high *HOXC6* expression was markedly linked to the advancement of malignant tumors, poor prognosis, and an immunoevasive environment in patients with CRC, with high presence of Tregs, CD8^+^ T-cells, neutrophils, and macrophages; declined levels of GZMB and PRF1; and elevated levels of PD-L1 and PD-1. This study demonstrated that high *HOXC6* expression was related to worse prognosis, promoting an immunoevasive environment and contributing to CD8^+^ T-cell dysfunction in patients diagnosed with CRC.

*HOXC6,* located on chromosome 12, has a crucial function in positional specification during the embryogenesis of multiple species, governing cellular differentiation. It is similar to other *HOX* family members [18]. However, aberrant expression of *HOXC6*, encompassing both upregulation and downregulation, may contribute to carcinogenesis [11]. *HOXC6* is considerably downregulated in the tissues of patients with serious ovarian cancers, accompanied by reduced levels in their serum [19]. In contrast, elevated *HOXC6* expression has been found to fuel cervical cancer evolution [20]. To our understanding, the correlation between the expression of *HOXC6* and its predictive importance in patients diagnosed with CRC has not been extensively investigated. Based on TCGA analysis and clinical validation, our study showed that *HOXC6* was excessively expressed in patients with CRC, and elevated expression of *HOXC6* was linked to the progression of malignancy and unfavorable survival outcomes in patients with CRC.

Nomograms are commonly used to determine cancer prognosis and inform clinical decision-making [21]. As a CRC prognostic nomogram based on *HOXC6* expression has not been previously reported, we constructed a prognostic nomogram to illustrate the relationship between six clinicopathological variables (*HOXC6* expression, age, CEA level, pathological stage, M stage, and KRAS status) and survival probabilities. After evaluating the C-index and calibration curve, the nomogram exhibited satisfactory performance in forecasting the likelihood of survival over 1, 3, and 5 years. Consequently, this nomogram holds potential for individualized prognostic prediction to improve the accuracy of high-risk patient identification. This result was validated within the Zhongshan Hospital cohort.

*HOXC6* is a critical transcription factor that regulates not only numerous *HOX* genes but also many other genes. A previous study identified SPARC, CST1 and KRT13 as the target genes of *HOXC6* in NSCLC. These genes are widely involved in regulating tumor evolution [22]. *HOXC6* directly regulates the gene expression of morphogenetic proteins and multiple growth factor receptors in prostate cancer [23]. In cervical cancer, *HOXC6* focuses on the promoter of the Bcl-2 gene, leading to the transformation of cervical epithelial cells and promoting tumor progression [20]. The above results indicate that *HOXC6* can regulate specific gene sets within different cellular environments to promote tumorigenesis. The *HOXC6* coregulatory proteins included in our study were *HOXA6*, *HOXB5*, *HOXB4*, *HOXB6*, *HOXA5*, *HOXA7*, *HOXC5*, *HOXC4*, and *HOXD4*. *HOX* genes have essential functions in numerous processes, including cell proliferation, angiogenesis, migration and inflammation. *HOXB3*, *HOXC8*, *HOXA13*, *HOXA7*, and others are dysregulated across numerous cancers and play a key role in malignant progression [[24], [25], [26], [27]]. *HOXB13* promotes tumor development by suppressing the cyclin kinase inhibitor p21 in prostate cancer [28]. *HOXA13* and *HOXB13* are also related to evading apoptosis [29,30]. Compared with normal ovarian tissue, the level of *HOXD1* in ovarian cancer tissue is elevated, suggesting that its activation may have a bearing on the dissemination of ovarian cancer [31]. *HOXA1* can activate cancer-related pathways and inflammatory processes in breast cancer cells [32]. Another study suggested that *HOXA4*, *HOXA5*, *HOXB6*, *HOXB4*, and *HOXC5* can regulate various metabolic processes, including oxidative phosphorylation, lipogenesis, fatty acid metabolism and glycolysis in tumors [33]. Consequently, these results indicated that *HOX* genes participate in the acquisition of malignant phenotypes and the development of tumors [10].

To elucidate the function of *HOXC6* in the development of CRC, we used KEGG and GSEA to identify biological pathways linked to *HOXC6*. Interestingly, GSEA revealed an augmented presence of the neutrophil degranulation pathway when the *HOXC6* phenotype was elevated. We also used ssGSEA to validate the increase in protumor cells (such as neutrophils, macrophages and Tregs) in the high-*HOXC6* expression group. Neutrophil mobilization of granules, a process known as degranulation, can occur at the plasma membrane to eliminate invading microorganisms [34]. A previous study proposed that neutrophils surround cancer cells in the bloodstream and transport them from the vascular system into tissues [35]. When migrating into the metastatic site, short-lived neutrophils undergo apoptosis and NETosis, triggering the further release of neutrophil constituents that create an immune-privileged site that helps cancer cells evade the immune system [36]. Upregulated *HOXC6* may thus contribute to the progression of malignancy in patients with CRC by promoting neutrophil degranulation. Notably, other immune-related signaling pathways were also associated with *HOXC6* expression and may also participate in the progression of cancer. These potential mechanisms are sophisticated and may interact within an integrated network.

Currently, it remains unclear how *HOXC6* participates in the development of an immunoevasive microenvironment and promotes tumorigenesis. To delve deeper into the immune-related mechanisms, we used IHC methods to detect the infiltration of a few immunocytes within the Zhongshan Hospital cohort. In the group with high *HOXC6* expression, the presence of macrophages, Treg cells, neutrophils, and CD8^+^ T-cells was increased. These findings are identical to those obtained through our ssGSEA. Tregs exert a tumor-promoting effect by suppressing adaptive antitumor immunity [37]. When the TME is rich in Treg cells, it can result in cytotoxic T-lymphocyte loss of function [38]. Tumor-associated macrophages are of vital importance in tumor initiation, growth, invasion, and distant dissemination and are considered to be the principal constituents of the TME. The density of macrophages within cancerous tissues is associated with adverse outcomes in most solid cancers [39]. Furthermore, immunocytes within the TME are key factors in the trajectory of tumor evolution. An increasing amount of proof backs the importance of immune cell distribution, composition, density, and functional status in forecasting the prognosis of tumor patients [[40], [41], [42]]. Our results show that the overexpression of *HOXC6* may promote cancer evolution and a worse outcome by affecting the regulation and recruitment of immunosuppressive cells within the TME.

In the TME, CD8^+^ T-cells are positive predictors and have long been regarded as antitumor cells on account of their power to directly attack tumors [43]. However, emerging evidence indicates that certain subtypes of CD8^+^ T-cells within tumors are related to poor clinical outcomes owing to their dysfunction [44]. We proved that the quantity of CD8^+^ T-cells in the high-*HOXC6* expression group was remarkably elevated, but the production of PRF and GZMB decreased, and the level of PD-L1 and PD-1 increased, leading to a dreadfully exhausted status and damaged immunological functioning in patients. In the TME, cancer cells bind to the PD-1 protein found on T lymphocytes through the PD-L1 ligand, making it impossible for T-cells recognize tumors and enabling cancer cells to evade immune system attacks [45]. The impact of tumors on immunocytes can result in T-cell incompetence or dysfunction, thereby promoting tumor evasion, progression, and treatment resistance [46]. Thus, we assumed that high *HOXC6* expression promotes an immunoevasive environment by upregulating the expression of immunosuppressive cells and immune checkpoint molecules, leading to T-cell dysfunction. Immune checkpoint inhibitors offer novel insights into CRC immunotherapy and have emerged as the most advanced immunotherapy in clinical application [47]. Due to tumor heterogeneity and immune escape, however, the effectiveness of immunotherapy in patients has been hindered; therefore, we need to find new targets. We observed an increase in PD-L1 and PD-1 in patients diagnosed with high *HOXC6* expression, suggesting the potential of *HOXC6* as a candidate biomarker for immunotherapy. Nonetheless, further research is required to validate this suggestion.

Our results suggest that high levels of *HOXC6* lead to CD8^+^ T-cell dysfunction and promote the formation of an immunoevasive TME, thereby accounting for the poor prognosis. Consistent with our study results, previous reports have indicated that the inhibition of CRC proliferation resulting from *HOXC6* knockdown may be regulated by the autophagy pathway, in which macrophages are also implicated [16]. In addition, CRC cells exhibiting high *HOXC6* expression fascinate an increase in CD8^+^ T-cells through the upregulation of chemokines that attract T-cells and molecules that regulate immune checkpoints. However, the downregulation of IFN-γ may deplete the performance of CD8^+^ T-cells [17]. Furthermore, Huang et al. [48] discovered that elevated levels of *HOXC6* in gliomas showed a positive association with increased stromal and immune scores, as well as elevated expression of various immune checkpoint genes (such as PD-L1 and CTLA-4). Although these studies used several bioinformatics methods to analyze the important role of upregulated *HOXC6* expression in tumor immunity, further cellular and animal studies are needed to confirm its role in immune dysfunction. We used two cohorts to confirm the expression of *HOXC6* in CRC and its relevance to malignant progression and worse outcome. We also validated the relationship between *HOXC6* and the immune-evasion microenvironment in CRC using IHC analysis. Previous studies have not reported the verification of these clinical samples. In the future, we plan to conduct more fundamental research to determine the specific mechanism by which *HOXC6* affects immune evasion.

Some studies have suggested that *HOXC6* is associated with immune dysfunction. In colon adenocarcinoma, a predictive hallmark according to the presence of CCKBR, *HOXC6*, and POU4F1 was discovered to be actively related to immune activity, microsatellite instability, gene expression of immune checkpoints, and poor sensitivity to chemotherapy [49]. This study was based on the TCGA and Gene Expression Omnibus (GEO) databases for bioinformatics analyses. Nonetheless, due to the absence of systematic verification for the predicted data, its applicability in clinical contexts must be verified. In CRC, the TME immune gene score system, consisting of SERPINE1, FABP4, SCG2, CALB2, and *HOXC6* genes, was intimately related to tumor evolution, infiltration of immunocytes, and poor response to immune checkpoint blockade (ICB). Among these molecules, *HOXC6* was the most significant. Analysis of several CRC databases revealed that the presence of *HOXC6* was actively related to T-cell incompetence and poor ICB outcomes. Among the immunosuppressive cells, *HOXC6* was highly expressed in myeloid-derived suppressor cells and cancer-associated fibroblasts. The “cytokine–cytokine receptor interaction” pathway was also remarkably concentrated in *HOXC6*. However, the predictive capacity of the model and the relationship among the five genes have not been verified in patients with CRC [50]. Another study suggested that *HOXC6* may affect the immune microenvironment and promote tumor evolution by adjusting the EMT signaling pathway in gliomas. Elevated expression of *HOXC6* has bearing on high infiltration of immunocytes, low tumor purity score, and elevated expression of immune checkpoint genes [48]. Their results were based on multiple bioinformatics analyses, but the concrete mechanism by which *HOXC6* regulates EMT and TME must be investigated. Another bioinformatics study on CRC indicated a strong correlation between increased HOXC6 expression and the cytokine pathway, as well as T-cell chemokine expression, infiltration of immunocytes and immune checkpoint expression [17]. Additional research is required to investigate the correlation between *HOXC6* and the TME in CRC. Currently, the correlation between HOXC6 and the TME has been inferred from bioinformatics studies through correlation analyses; in-depth research on the underlying mechanism or causality demonstrations has been limited. In our study, we confirmed that high HOXC6 expression facilitated an immunoevasive environment through the upregulation of the expression of immunosuppressive cells and immune checkpoints, resulting in T-cell dysfunction in the Zhongshan Hospital cohort. Our study offers more clinical verification than previous bioinformatics studies, although further investigation is required to elucidate the effect of *HOXC6* on tumor immunity.

Numerous researches have proposed that *HOX* genes are regarded as dormant indicators and treatment targets in many malignancies. In a prospective multicenter study, a risk score was constructed by combining urine expression levels of *HOXC6* and DLX1 mRNA with conventional hazard factors. This score precisely detected high-grade prostate cancer, thus enhancing the diagnosis and therapeutic management of patients with prostate cancer and reducing unnecessary prostate biopsies [51]. Recently, a clinical trial found that low-dose gemcitabine induces hypomethylation of CpG islands within the *HOXA10* and *HOXA11* genes, restoring sensitivity to carboplatin and improving the survival rate in patients diagnosed with ovarian cancer [52]. Studies conducted in laboratory settings and living organisms have demonstrated that HXR9 can cut off the interplay between many different *HOX* proteins and their cofactor PBX, leading to transcriptional changes in potential target genes and ultimately inhibiting tumor evolution. Targeting the *HOX*/PBX interaction may be an efficacious method for treating esophageal squamous cell carcinoma [53]. Similar results have been reported for other tumor types [[54], [55], [56]] but not for CRC. Using connectivity mapping and cell experiments, Li et al. [57] proved that vincristine could reverse the CD133/*HOX* genes/LIM2 signatures expression within gliomas. The results indicated the coexpression of CD133 and *HOX*, suggesting that increased CD133 and *HOX* expression could serve as predictive markers for vincristine sensitivity. Although numerous studies have suggested *HOX* as a therapeutic target for various malignant tumor types, reports regarding its role in CRC are lacking.

Some studies have examined whether *HOXC6* expression could be used to assess prognosis and sensitivity to treatment in CRC. Ji et al. [16] pressed that downregulated expression of *HOXC6* inhibits CRC evolution both in vivo and in vitro, mainly through the inhibition of the autophagy pathway. They pointed out that *HOXC6* may be a potential therapeutic marker, although clinical verification is lacking. A basic research study showed that TrkB/C activation leads to subsequent activation of MEK/ERK signaling pathway, promoting the activation of ADAM8 mediated by *HOXC6* and inducing the metastasis of colon cancer cells that are resistant to chemotherapy. The researchers speculated that targeting *HOXC6*, TrkB/C and ADAM8 might be a novel approach for treating patients with drug-resistant colon cancer; however, this must be verified in the future [58]. A bioinformatics study suggested that *HOXC6* is likely to be a latent target immunotherapy of CRC, although it lacked support from prospective or mechanistic research [17]. Another study suggested that overexpression of *HOXC6* in right-sided colon cancer could activate the Wnt/β-catenin signaling pathway, inhibit the secretion of DKK1, induce intestinal epithelial cell transformation, and promote tumor cell migration. It was confirmed that silencing *HOXC6* can increase the vulnerability of HCT116 and HT29 cells to irinotecan. It is anticipated that *HOXC6* will become a target for therapy in CRC, thereby expanding the utility of irinotecan in CRC treatment [59]. Evidently, *HOXC6* is a latent indicator and treatment target for CRC; however, support from targeted therapy or clinical studies remains imperative.

Several studies have declared that other potential biomarkers are related to the immunoevasive microenvironment of CRC. Lee et al. [60] identified that S100A14 inhibits STAT3-mediated PD-1 expression and the phenotype of tumor stem cells, promotes CD8^+^ T-cell-mediated cytotoxicity, inhibits immune evasion, and restores chemosensitivity. Thus, targeting S100A14 is likely an effective strategy for preventing CRC progression, and S100A14 could be regarded as a promising indicator for anti-PD-L1 immunotherapy and chemotherapy. Yu et al. [61] found that INHBA is grossly coexpressed alongside T-cell biomarkers and immune checkpoints, serving as a new means of regulating immune evasion mechanisms in CRC cells. The finding indicated the potential utility of INHBA as a prognostic factor in CRC. Rabinovitch et al. [62] found that galectin-1 (Gal-1) enhances the quantity and effectiveness of CD8^+^ regulatory T-cells and promotes immune evasion mechanisms in CRC cells. Therefore, Gal-1 can regulate immune activity and improve the prognosis of patients with CRC. Gal-1 targeting may be a potential immunotherapeutic strategy. These results were obtained through basic research or bioinformatics studies, and validations were only performed at the clinical sample level. Future studies should focus on targeted therapy and expanded clinical studies to examine their applicability within the context of CRC.

To date, two markers with clinical relevance for CRC prognosis have been identified: defective DNA mismatch repair (dMMR) status [[63], [64], [65]] and the V600E BRAF mutation [66]. The former has been related to better prognosis in patients diagnosed with stage II or III colon cancer who did not have fluorouracil-based treatment, while the latter is related to a worse outcome. When compared with recognized prognostic biomarkers, such as dMMR status or BRAF status in CRC, which have been demonstrated in phase III clinical studies with elements such as randomization, large sample size, robust data, and high credibility [[64], [65], [66]], the prospect of *HOXC6* as a promising biomarker for CRC must be demonstrated in additional clinical and mechanistic studies.

The strength of this study was that it comprehensively investigated the role of *HOXC6* in CRC using TCGA data and validated the relevance between *HOXC6* expression and the TME using clinical data. To our understanding, the relevance between *HOXC6* level and the immunoevasive microenvironment has not been sufficiently elucidated. The upregulation of *HOXC6* leads to immune evasion within the TME, and it is likely that HOXC6 can act as an indicator for identifying patients suitable for immunotherapeutic interventions. However, further investigation is required to fully ascertain the exact correlation between *HOXC6* and the response to anticancer treatment, a task that requires exploration within a large cohort of CRC cases.

However, this study has certain limitations; for instance, our sample size was relatively small. In addition, our data were procured from a single database (TCGA), and the results may be more convincing if comparisons were made with other databases. Furthermore, information in the dataset about treatment and response was incomplete, and we could not estimate the effect of *HOXC6* during the treatment of CRC. Therefore, the substantiation of our conclusions requires the use of a larger sample size and the inclusion of supplementary external cohorts. Moreover, the underlying mechanism facilitating immune evasion associated with high *HOXC6* expression in patients diagnosed with CRC remains unclear, warranting a more extensive study.

## 4 Conclusions

Elevated level of *HOXC6* in patients diagnosed with CRC is linked to poorer prognosis and the promotion of an immunoevasive TME. Although further investigations are needed, our study shows that *HOXC6* could potentially become an indicator to predict the outcome of patients diagnosed with CRC.

## 5 Methods and materials

### 5.1 Data obtained from RNA sequencing and subsequent analysis using bioinformatics

Using the R package “TCGAbiolinks”, we acquired the clinical records and gene expression data of 619 patients with CRC (workflow type: HTSeq-FPKM) from TCGA. UCSC XENA (https://xenabrowser.net/datapages/?hub=https://toil.xenahubs.net:443) provided TCGA and GTEx TPM format RNAseq data, which were intensively handled through the Toil process. Instances of healthy colorectal specimens and cases where the OS time was less than 30 days were eliminated from the study. Subsequently, HTSeq-FPKM data were converted to transcripts per million reads (TPM) for further studies. The characteristics of the patients (namely, TNM stage, pathological stage, sex, CEA level, neoplasm type, presence of colon polyps, history of colon polyps, KRAS status, BRAF status, TP53 status, and age) were took notes. Missing values were assigned to clinical characteristics that were unusable or unknown.

### 5.2 PPI network

We utilized the STRING database (https://cn.string-db.org) to build a PPI meshwork and selected genes with scores >0.4 to construct a network model.

### 5.3 GO and KEGG pathway

GO analysis is an extensively applied approach within functional enrichment studies. This approach can generate data interrelated with biological processes, molecular functions, and cellular components. KEGG is a data library designed for the systematic analysis of genetic functions, connecting genomic information with meticulously organized biologic functional information.

### 5.4 GSEA

In our study, GSEA was conducted utilizing the R package cluster analysis (3.8.0) to clarify the major pathway discrepancies between groups exhibiting high and low expression of HOXC6. Each analysis involved 1000 gene set permutations. The expression of *HOXC6* served as the phenotypic marker. Pathway enrichment was analyzed according to the adjusted p value (<0.05) and FDG q-value (<0.25).

### 5.5 Analysis of immune infiltration using ssGSEA

We analyzed the presence of 24 immunocytes in CRC samples using ssGSEA (applying the GSVA package in R [3.6.3]). The ssGSEA method categorizes sets of marker genes with shared biological functions, chromosomal assignment, and physiological regulation into a singular sample. Based on the gene expression profile of each tumor sample, the quantification of the relative enrichment fraction of every immunocyte was determined, taking into account the characteristic genes of the 24 immunocytes mentioned in the literature.

### 5.6 Establishing the prediction model

We predicted the OS of patients diagnosed with CRC using uni- and multivariate Cox analyses. Clinical pathological characteristics were combined into a model to structure a clinical prognostic nomogram. We used the Harrell consistency (C) index to evaluate the performance of the nomogram. Furthermore, a correction graph was drawn to assess the performance of the nomogram.

### 5.7 Individuals and CRC tissue specimens

Between the dates of 2009/1/1 and 2010/12/30, 232 patients who had experienced CRC surgery were recruited in the cohort from Zhongshan Hospital. The cohort from the Shanghai Cancer Center consisted of 344 patients who underwent CRC surgery between 2011/1/1 and 2012/12/30. However, 32 patients from the Zhongshan Hospital cohort and 44 patients from the Shanghai Cancer Center cohort were excluded due to incomplete survival outcomes or clinicopathological data, benign tumors/carcinomas in situ, emergency surgeries, or a history of malignant cancer. Finally, 200 and 300 patients from Zhongshan Hospital and the Shanghai Cancer Center, respectively, were successfully included in this research. The period of follow-up concluded on 2020/12/31. The recorded characteristics included sex, age, tumor location, tumor differentiation, tumor histology, surgical margin positivity, nerve invasion, number of cancer nodules ≥1, infiltrating lymph nodes >12, and pathological stage. We conducted analyses on both cancerous and noncancerous tissues. Noncancerous tissue refers to tissues located 2 cm away from the tumor focus. The use of this clinical record was authorized by the Ethics Committee of Shanghai Cancer Center (IRB2105235-6) and Zhongshan Hospital (B2022-068R2). All the patients participating this research provided informed consent.

### 5.8 Western blotting

Ice-cold lysis buffer was added to the tissue and homogenized using an electric homogenizer. After being agitated at a temperature of 4 °C for a duration of 2 h, the contents were subjected to centrifugation, and the resulting supernatant, which contained protein, was collected. The content of total protein was determined using the BCA protein analytical reagent. After the samples were added, the voltage during electrophoresis was 80V. Subsequently, upon the marker's entry into the separation gel, the voltage could be modified to 120V. Electrophoresis could be concluded by allowing it to run to the bottom of the gel, after which the membrane can be transferred. After transferring the membrane, it was immersed in a blocking solution consisting of 5 % skim milk powder and blocked for approximately 1 h at a temperature of 22–24 °C. The membrane was then transferred to a new incubator, where the primary antibody was diluted and added. The membrane was then incubated at 4 °C overnight. The secondary antibody was appropriately diluted with PBST and incubated for 1 h at 22–24 °C. Azure Radiance Q reagent (Azure Biosystems, CA, United States) was then prepared. The excess wash buffer was drained from the blot and then placed on a clean and dry surface. The working solution of the substrate was then poured onto the membrane and allowed to incubate for 5 min for exposure. Anti-*HOXC6* antibodies (ab151575) were purchased from the manufacturer (Abcam, Cambridge, UK), with β-actin serving as the loading control.

### 5.9 RNA separation and RT‒qPCR

We collected total RNA utilizing TRIzol reagent (Invitrogen, Waltham, MA, USA). SYBR Green Supermix (Thermo Fisher, #1176202K) and a PrimeScript RT kit (Takara, Shiga, Japan) were used to prepare cDNA via reverse transcription. We employed an ABI 7900HT real-time PCR system (Applied Biosystems, Carlsbad, CA, USA) to identify the expression of genes via quantitative reverse transcription PCR. The relative levels of transcription were estimated using the ΔΔCt technique. The sequences were 5′-GGAGCGAGATCCCTCCAAAAT-3′ and 5′-GGCTGTTGTCATACTTCTCATGG-3′ for *GAPDH* (human) primers and 5′-ACAGACCTCAATCGCTCAGGA-3′ and 5′-AGGGGTAAATCTGGATACTGGC-3′ for *HOXC6* (human) primers.

### 5.10 IHC staining

Paraffin-embedded tissues were dewaxed and cleaned. The tissue slices were soaked in a citric acid antigen repair buffer (pH 6.0) at medium heat for 10 min until boiling, followed by a 10-min cool-down period and then 7 min of medium-low heat. We handled the slices using a solution of 3 % hydrogen peroxide (where hydrogen peroxide is mixed with pure water in a ratio of 1:9) and cultured them in darkness at 22–24 °C. To overlap the tissue evenly, 3 % BSA solution was added. After adding the primary antibody, the slices were incubated at 4 °C overnight. A 50-min incubation at room temperature was performed after introducing the secondary antibody. Once the slices were partially dried, a freshly prepared DAB chromogenic solution was dropped into the circle. Nuclei were stained using Harris hematoxylin. After dehydrating and sealing the sections, they were examined microscopically, and then images were acquired and analyzed. The staining score was calculated by two pathologists. The concentrations of CD8^+^ T-cells, Foxp3^+^ Tregs, CD68^+^ macrophages, CD66b^+^ neutrophils, granzyme B (GZMB), perforin (PRF1), programmed cell death-ligand 1 (PD-L1), and programmed cell death protein 1 (PD-1) were recorded by randomly counting Six high-power fields (HPFs, 200X magnification), with each field being counted three times. Supplementary Table 9 shows the immunohistochemical antibodies used in this study.

### 5.11 Statistical analysis

We conducted all statistical analyses using IBM SPSS Statistics 25.0 (SPSS Corp., Armonk, NY, USA) and R (v.3.6.0) (R Foundation for Statistical Computing, Austria). We analyzed the level of *HOXC6* in paired and unpaired samples using the Wilcoxon signed-rank test and Wilcoxon rank-sum test, respectively. To assess the relevance between *HOXC6* expression and clinical pathological features, we used the Kruskal–Wallis test, logistic regression, and Wilcoxon signed-rank test. The cutoff value was determined according to the median expression of *HOXC6*. Prognostic factors were examined adopting the Kaplan–Meier method and Cox regression analyses. The impacts of *HOXC6* and other clinical features on survival were studied by adopting both univariate and multivariate Cox analyses. To examine the relevance between *HOXC6* expression and immunocytes, we employed the Spearman correlation test. We employed the Wilcoxon rank-sum test to examine the variation in immunocyte infiltration levels between the high- and low-*HOXC6* expression groups. During the clinical verification stage, we employed the Mann–Whitney *U* test to calculate the discrepancies between two sets of continuous variables. Significance was established for all tests listed hereafter: *P < 0.05, **P < 0.01, and ***P < 0.001.

## Data availability

Our data was downloaded from UCSC XENA (https://xenabrowser.net/datapages/?hub=https://toil.xenahubs.net:443). Source data for all graphs in this manuscript are provided in the article and supplemental materials. If reasonably requested, any other data of this study can be obtained from the authors.

## Ethics approval and consent to participate

The ethics committee of 10.13039/501100010108Zhongshan Hospital, 10.13039/501100003347Fudan University (B2022-068R2) and Shanghai Cancer Center, 10.13039/501100003347Fudan University (IRB2105235-6) granted authorization for our study. Before the study, all the individuals involved in the study provided their informed consent by signing the necessary documents.

## Funding

Our study was supported by the 10.13039/501100001809National Natural Science Foundation of China (Nos. 82002538, 82372502); 10.13039/100007219Natural Science Foundation of Shanghai (No. 23ZR1462800); 10.13039/100007219Natural Science Foundation of Shanghai Municipal Commission of Science and Technology (No. 23ZR1411400); 10.13039/501100003399Science and Technology Commission of Shanghai Municipality-Medical Innovation Research Special Project (23Y11902300); 10.13039/501100010108Zhongshan Hospital Clinical Research Special Funding (ZSLCYJ202346).

## CRediT authorship contribution statement

**Meilin Weng:** Conceptualization, Data curation, Formal analysis, Funding acquisition, Investigation, Methodology, Supervision, Validation, Visualization, Writing – original draft, Writing – review & editing. **Yuling Lai:** Conceptualization, Formal analysis, Methodology, Writing – review & editing. **Xiaodong Ge:** Investigation, Methodology, Validation. **Wenchao Gu:** Investigation, Methodology, Validation. **Xixue Zhang:** Conceptualization, Supervision, Writing – review & editing. **Lihong Li:** Conceptualization, Visualization, Writing – review & editing. **Minli Sun:** Conceptualization, Funding acquisition, Writing – review & editing.

## Declaration of Generative AI and AI-assisted technologies in the writing process

We didn't employ AI and AI assisted technologies in the writing process.

## Declaration of competing interest

The authors declare that they have no known competing financial interests or personal relationships that could have appeared to influence the work reported in this paper.

## Figures and Tables

**figs1:** 

**figs2:** 

**figs3:** 

**figs4:** 
